This article has been retracted.

# Probiotic Supplement Preparation Relieves Test Anxiety by Regulating Intestinal Microbiota in College Students

**DOI:** 10.1155/2021/5597401

**Published:** 2021-04-20

**Authors:** Qi Qin, Hui Liu, Yulu Yang, Yifei Wang, Chaofei Xia, Puyuan Tian, Jing Wei, Shengjie Li, Tingtao Chen

**Affiliations:** National Engineering Research Center for Bioengineering Drugs and the Technologies, Institute of Translational Medicine, Nanchang University, Nanchang, Jiangxi Province 330031, China

## Abstract

Test anxiety creates barriers to learning and performance, which further affects students' social, behavioural, and emotional development. Currently, the medication to treat test anxiety has not been reported yet. Here, we enrolled 120 students to evaluate the effect of probiotic supplement preparation (PSP) on test anxiety from the aspect of the intestinal microbiota. We found that the intake of PSP alleviated the symptoms of depression and anxiety in students with test anxiety by evaluating their mental state using the Hamilton Depression Rating Scale and Hamilton Anxiety Scale. High-throughput sequencing results indicated that the consumption of PSP increased the abundance of *Streptococcus* and *Akkermansia* that was lowered by the anxiety state in the intestinal microbiota of students. Meanwhile, taking PSP reduced the level of intestinal pathogens of *Fusobacterium* and *Clostridium* as well. In conclusion, our work shows that PSP can reduce test anxiety and restore the disturbed microbiota to the standard level in Chinese college students, rendering the use of PSP a promising strategy for test anxiety.

## 1. Introduction

Test anxiety is a physiological symptom that is combined with the fear of failure, dread, catastrophizing, and worrying before and during a test, which negatively affects the social, behavioural, and emotional development of students and their feelings about school and themselves [1]. It is a common and potentially serious problem among college students and affects about 20-40% of all students, with a higher prevalence in the students with learning disabilities [1, 2]. A variety of interventions and strategies have been proven beneficial to relieve test anxiety, e.g., using student-friendly tests, enhancing accessibility, fostering motivation, and collaborating with family members and other professionals [1]. Enacting habits to reduce stress, such as exercise, proper nutrition, improving sleep, studying without fear, and meditation, are recommended for treating test anxiety as well [2]. However, the medication to treat test anxiety has not been reported yet.

Growing evidence has explored the potential influence of microbiota on the brain-gut axis in health and disease, including nutrition, immunity, host physiology, and brain development [3, 4]. It has also been suggested that the intestinal microbiota is involved in the modulation of behaviour in stress-related disorders [3, 5, 6]. Studies have indicated that some probiotics can produce neurotransmitters and neuromodulators (e.g., *γ*-aminobutyric acid, norepinephrine, and dopamine) to modulate opioid and cannabinoid receptors in the gut epithelium and relieve depression and anxiety [7–10].

Although many researchers have indicated the link between intestinal microbiota and mental disorders, little work has been done to evaluate the effect of probiotics on test anxiety in students and their influence on the intestinal microbiota of students. In the present study, the probiotic supplement preparation (PSP) of Hengxin probiotics was used to test the effect of probiotics on test anxiety in Chinese college students.

## 2. Materials and Methods

### 2.1. Ethics Statement

All subjects gave their informed consent for inclusion before they participated in the study. The study was conducted in accordance with the Declaration of Helsinki, and the protocol was approved by the Ethics Committee of the Second Affiliated Hospital of Nanchang University (Examination and approval no. is Review [2019] No. (039)).

### 2.2. Study Groups and Sampling

PSP of Hengxin probiotics was a gift from Harbin Meihua Biotechnology Co., Ltd. (Harbin, Heilongjiang, P.R. China), containing 1.2 × 10^10^ CFU of *Bifidobacterium longum* subsp. *Longum* BAMA-B05/Bau-B1024, 1.9 × 10^10^ CFU of *B. lactis* BAMA-B06/Bau-B0111, 1.5 × 10^10^ CFU of *B. adolescentis*, 3.2 × 10^9^ CFU of *Streptococcus thermophiles*, 4.6 × 10^9^ CFU of *Lactobacillus acidophilus*, and 3.0 × 10^9^ CFU of *L. delbrueckii* subsp. *bulgaricus* per 100 grams of the granule's product, respectively, with a total number of over 10^9^ CFU of viable bacterial count per package. The product qualities were also evaluated by the total viable count method and 16S rDNA sequencing before using it.

A total of 300 college students (aged between 18 and 24 years) were enrolled randomly in this study, and 43 of them dropped out due to personal reasons. And then, the eligibility of the rest of the students was assessed by interviewing them about their daily behaviours and health conditions. As a result, 137 students were excluded due to the following reasons, e.g., smoking, drinking, taking antibiotics regularly, and obese and flu sufferers were ruled out as well. Finally, 120 members were selected to respond to questionnaires assessing the depressive and anxiety symptoms at Nanchang University (Table S1). Sixty students without test anxiety were allocated to the healthy group and used as the control one (H group, taking the same package with no probiotics as placebo). The other sixty students with test anxiety were assigned as the treatment group and divided into two subgroups, named BP group meaning before taking the PSP and AP group which took PSP for 15 consecutive days (twice per day, and approximately 12-hour set time between two intakes) (Figure 1). The random fecal samples from the H group (*n* = 30), BP (*n* = 30), and AP (*n* = 30) groups were collected by a stool sampling tube according to the manufacturer's introduction. All the fecal samples were stored at -80°C immediately for DNA extraction [11].

### 2.3. Depressive and Anxiety Symptoms Analysis

The depressive symptoms of students were evaluated by trained psychiatrists using the Chinese version of the 17-item Hamilton Depression Rating Scale (HAMD-17). The severity of the depressive symptoms was classified using the following severity range for the HAMD score: normal (0–7), mild depression (8–16), moderate depression (17–23), and severe depression (>23). The anxiety symptoms were evaluated using the Chinese version of the 14-item Hamilton Anxiety Scale (HAMA-14), and anxiety symptom severity was classified by the following severity range for the HAMA score: normal (0–7), mild or probable anxiety (8–14), moderate or definite anxiety (15–21), and severe anxiety (≥22) [12].

### 2.4. Genomic DNA Extraction and High-Throughput Sequencing

For the DNA extraction of faeces, a combination of the bead-beating method and Genomic DNA kits (Tiangen Biotech Co., Ltd., Beijing, China) were applied [13]. The concentration and quality of the purified DNA were determined at spectrophotometer (NanoDrop, Thermo Fisher Scientific, Inc., USA). Then, primers 515F/806R (5′-GTGCCAGCMGCCGCGGTAA-3′ and 5′-GGACTACVSGGGTATCTAAT-3′, respectively) were used to amplify the V4 region of the 16S rDNA genes in each sample, and these PCR products were sequenced with an Illumina HiSeq 2000 platform [14]. The raw reads were deposited in the Sequence Read Archive (SRA) database of NCBI (PRJNA530283).

### 2.5. Bioinformatics and Multivariate Statistics

FLASH software was used to map overlapped reads (http://ccb.jhu.edu/software/FALSJ/), and low-quality sequences were eliminated by QIIME (v1.8.0, http://qiime.org/) according to the following criteria: (a) raw reads shorter than 160 bp and contained N base; (b) >1 mismatches in the 5′-primer; (c) sequences with more than eight continuous same bases. The obtained sequences were checked by UPARSE package (v 5.2.236) and removed the chimeric ones. Sequences with ≥97% similarity were performed as the same operational taxonomic units (OTUs) using an open-reference OTU picking protocol. The relative abundance of each OTU was assigned as a proportion of the sum of sequences of each sample. The *α*-diversity (within samples, indexes of observed OTUs, Chao1, Shannon) and *β*-diversity (among samples, PCA, NMDS) were calculated by QIIME software as well.

### 2.6. Statistical Analysis

Statistical analysis was performed using Prism software version 7.0 (GraphPad Software, San Diego, CA, USA). Data was shown as the mean ± SD. Statistical significance was analysed using a one-way analysis of variance (ANOVA) followed by Tukey's multiple comparison test. Error probabilities of *p* < 0.05 were considered statistically significant.

## 3. Results

### 3.1. PSP Alleviated Test Anxiety

First, we evaluated the ability of the PSP to improve the mental state of students. As shown in Figure 2, our results indicated that exam pressure significantly increased students' depression (BP) compared with the students without test anxiety (H) (10.15 vs. 1.92, *p* < 0.01), while the administration of the PSP markedly alleviated students' depression from 10.15 (BP) to 3.87 (AP) (*p* < 0.01) (Figure 2(a)). Similarly, the anxiety scale in the BP group was as high as 10.85, while probiotics significantly reduced the anxiety in the AP group to 3.93 (*p* < 0.01) (Figure 2(b)).

### 3.2. PSP Had Little Effects on the Microbial Diversity

To evaluate the effect of PSP on microbial diversity, we collected and assessed every 30 fecal samples from the H, BP, and AP groups. It seemed that the PSP had little impact on the Shannon index (5.69, 5.54, and 5.84) and Chao1 index (662, 657, and 692.6) among the H, BP, and AP groups, respectively (Figures 3(a) and 3(b)). The Venn diagram results indicated that 86.76% (3051/3517) of the bacteria were common among the H, BP, and AP groups, yet 18 unique bacteria were found existing in the BP samples (Figure 3(c) and Table S2). Moreover, the PCA and NMDS results indicated that the samples in the H group, BP, and AP groups clustered together (Figure 3(d) and Figure S1).

### 3.3. Effects of PSP on the Microbial Community at the Phylum Level

As shown in Figure 4, data for the top 20 microorganism populations at the phylum level were analysed. *Firmicutes*, *Bacteroidetes*, *Actinobacteria*, and *Proteobacteria* constituted the four most common dominant phyla in the H group (0.58, 0.21, 0.15, and 0.05, respectively), BP (0.64, 0.18, 0.10, and 0.05, respectively) group, and AP (0.63, 0.18, 0.08, and 0.07, respectively) group, which accounted for 0.99, 0.97, and 0.97 of the total sequencing number in these three groups, respectively (Figure 4(a)). Then, we further evaluated the relative abundance of *Firmicutes*, *Bacteroidetes*, and *Actinobacteria* in groups H, BP, and AP. Results suggested that the administration of PSP had little effect on the composition of *Firmicutes* and *Bacteroidetes*, while it seemed that the test anxiety could significantly reduce the abundance of *Actinobacteria* (Figures 4(b)–4(d)). Therefore, it seems that the administration of probiotics has little effect on the microbiota at the phylum level.

### 3.4. Effects of PSP on the Microbial Community at the Genus Level

Then, the top 20 genera were analysed. *Bifidobacterium*, *Bacteroides*, *Faecalibacterium*, *Ruminococcus*, *Prevotella*, and *Clostridium* accounted for the dominant bacteria in most samples in the H, BP, and AP groups (Figure 5(a)). To better evaluate the effect of PSP on specific genera, *Fusobacterium*, *Clostridium*, *Prevotella*, *Streptococcus*, and *Akkermansia* were further studied. Our results indicated that students with test anxiety had an increased abundance of the pathogens of *Fusobacterium* (0.00008 vs. 0.01443) and *Clostridium* (0.021 vs. 0.034) and a reduced abundance of *Prevotella* and *Streptococcus* (0.0217 vs. 0.0129), while taking PSP obviously reduced the abundance of *Fusobacterium* (0.01443 vs. 0.0001) and *Clostridium* (0.034 vs. 0.023) and enhanced that of *Streptococcus* (0.0129 vs. 0.0283) and *Akkermansia* (0.0076 vs. 0.0219) (Figures 5(b)–5(f)).

## 4. Discussion

Test anxiety is a type of performance anxiety in which people experience extreme distress and anxiety when tested, resulting in impaired learning and reduced performance on tests. Test anxiety has dramatically influenced studies and lives among students in elementary school, middle school, and high school. Here, we evaluated the effectiveness of a multiple probiotics granules product that has been approved by the State Food and Drug Administration of China as a kind of health-care food with the function of enhancing immunity and defecating, on the alleviation of the test pressure. As we know, when students suffer from test anxiety, they feel helpless and anxious, which significantly affects their study, sleep, and diet, and the unhealthy diet and lifestyle, in turn, increases the test anxiety in students.

Research studies have indicated that probiotics have benefits in reducing gastrointestinal discomfort, improving immune health, and relieving constipation [15]. Some work has suggested that people who consume probiotics maintain a healthy balance between anti- and proinflammatory responses, which exerts the potential benefits of gut bacteria on brain health [16]. Kim and Shin indicated that probiotic food consumption has beneficial sound effects on depression [15], and the work performed by Pinto-Sanchez et al. also reported that probiotics successfully reduced depression and increased the quality of life in patients with irritable bowel syndrome (IBS) [6]. As test anxiety is a mild psychological condition, we hypothesized that a probiotic supplement is sufficient to enhance the mental state of students with test anxiety.

In support of our hypothesis, the consumption of PSP alleviated the depression scale and anxiety scale of students. Many reports have indicated that probiotics could reduce various neurological diseases (e.g., Parkinson's disease and Alzheimer's disease) and anxiety caused by illness or depression [6, 16–19]. Thus, it is easy to understand that probiotics will exert a much better effect on the mild psychological condition of test anxiety. In the next step, we further evaluated the impact of probiotics on intestinal microbial diversity, and it seemed that the short period of probiotic consumption reduced the individual differences among students in the AP group compared with students in the H and BP groups, and slightly increased the Shannon index and Chao1 index.

Then, we compared the microbial composition among the H, BP, and AP groups. At the phylum level, test anxiety and probiotics hardly influenced the abundance of *Firmicutes* and *Bacteroidetes*, while could reduce plenty of *Actinobacteria*, and probiotic consumption failed to bring it back to normal levels. *Actinobacteria* is a phylum of gram-positive bacteria with great economic importance, which can produce bioactive metabolites that are useful in human medicine, such as antibacterials, antifungals, antivirals, antithrombotics, immune modifiers, antitumor drugs, and enzyme inhibitors [20]. At the genus level, test anxiety enhanced the abundance of the pathogens *Fusobacterium* and *Clostridium* and reduced the abundance of *Streptococcus*. However, probiotic administration for 15 days could increase the levels of *Streptococcus* and *Akkermansia*, while reducing the levels of the pathogens *Fusobacterium* and *Clostridium* (Figure 4). As pathogens, *Fusobacterium* and *Clostridium* have been reported to have strong connections with various diseases (e.g., cancers, Alzheimer's disease, and Parkinson's disease), and their overgrowth significantly enhances the deterioration of conditions [21–24]. As probiotics, *Akkermansia*, and *Streptococcus* have been reported to possess benefits in cases of IBS, cancers, infection, obesity, diabetes, and inflammation [25–28]. Although the intestinal microbiota is associated with stress-related disorders, we should not just diagnose the status of anxiety from the aspect of gut microbiota since it would be affected frequently by some other factors, e.g., food habit, drug abuse, and individual differences. But probiotics consumption could be regarded as a kind of treatment and intervention method for relieving human anxiety via modulating the balance of gut micriobiota in the future [29].

## 5. Conclusion

In the present study, we evaluated the anti-test anxiety effects of Hengxin probiotics. We found that this PSP could significantly reduce test anxiety by reducing the number of pathogens and increasing of probiotics. However, this study has some limitations, e.g., the lack of a group with test anxiety but taking no probiotics (due to the unwillingness of students to take excipients). Additionally, it would have been more informative if some neurotransmitters and metabolites in the faeces were monitored. This is the first study that probiotics are suggested to associate with lower test anxiety in Chinese college student significantly. Our findings provide meaningful information that PSP might play a role in lowering the risk of depression and anxiety in Chinese students.

## Figures and Tables

**Figure 1:** Students included in this study. The trial enrolled 300 students, and 120 students (aged between 18 and 24 years) were finally recruited based on the evaluation of depressive and anxiety symptoms at Nanchang University.

**Figure 2:** PSP improves the mental state of students suffering test anxiety. (a) PSP alleviated students' depression by reducing Hamilton Depression Scale. (b) PSP relaxed the anxiety scale by reducing Hamilton Anxiety Scale. H: students without test anxiety (*n* = 60); BP: students before taking PSP (*n* = 60); AP: students after taking the PSP (*n* = 60). ^∗∗^*p* < 0.01.

**Figure 3:** Effects of PSP on the intestinal microbial diversity in students. (a) Shannon index of fecal microbiota. (b) Chao1 index of fecal microbiota. (c) Venn diagram of fecal bacteria species. (d) PCA analysis of shared genera among microbiomes in the H, BP, and AP groups. H: students without test anxiety (*n* = 30); BP: students before taking PSP (*n* = 30); AP: students after taking PSP (*n* = 30).

**Figure 4:** PSP has little effect on fecal microbiota composition at the phylum level. (a) The relative abundance of the top 20 bacteriophyta. (b) The relative abundance of *Actinobacteria*, (c) *Bacteroidetes*, and (d) *Firmicutes*. H: students without test anxiety; BP: students before taking PSP; AP: students after taking PSP. ^∗^*p* < 0.05, ^∗∗^*p* < 0.01.

**Figure 5:** PSP enhances the relative abundance probiotics in anxious students. (a) The relative abundance of the top 20 microbes. (b) The relative abundance of *Fusobacterium*, (c) *Clostridium*, (d) *Prevotella*, (e) *Streptococcus*, and (f) *Akkermansia*. H: students without test anxiety; BP: students before taking PSP; AP: students after taking PSP.

## Data Availability

The datasets used and/or analysed during the present study are available from the corresponding author on reasonable request.

## Supplementary Materials

Supplementary 1 Figure S1: Nonmetric Multidimensional Scaling (NMDS) analysis of shared genera among microbiomes in the H, BP, and AP groups.

Supplementary 2 Table S1: baseline patient demographics and characteristics. Table S2: the unique bacteria existed in the test anxious students before taking PSP.
